This article has been retracted.

# Research on Computer-Aided Product Design Technology

**DOI:** 10.1155/2022/7770690

**Published:** 2022-07-18

**Authors:** Wei Song

**Affiliations:** School of Fine Arts, Linyi University, Linyi, Shandong 276000, China

## Abstract

As globalization picks up speed, product innovation—the driving force behind business growth and market competition—becomes increasingly important for advancing product design technology. Computer-aided technology is one of the key components of product design, including issues with scientific analysis, creative thinking, problem-solving, and handling conflicts. Product design technology is gaining more and more attention. Computer-aided technology is now a trendy topic that is being studied by many academics due to the quick growth of computer technology. However, most of them focus on the product information model and solution and do not start from the technical methods and innovation of product design, resulting in many problems in the later solution and information description. Therefore, this paper studies product technology problems based on computer-aided technology and briefly explains the CAI technology-driven technology and the establishment of integrated process model. In this model, the assembly information model diagram is constructed to analyze the conflicts and problems in the assembly model, and then, the CAI-driven integrated innovation technology is called to complete the assembly model design. Conflicts in the assembly design can be minimized by using this paradigm. Finally, the qualitative examination of product design reveals that brainstorming is the process that uses the least amount of energy. The shafting assembly system is reviewed and examined at the same time, and the assembly accuracy accounts for the highest 35 percent of the system, completely indicating the extraordinary impact of computer-aided product design.

## 1. Introduction

Generally, computers are used in almost every domain of life starting from the very basic to the complication and crucial task or organizations. These computers are used for the smooth running of the various business and are used as a handle, i.e., which has the capacity to ease task of the individuals and enable and timely and quickly processing of the applications. However, as the business processes are expended with the passage of time, there is always a need for the dedication systems which are specifically developed for the task which are under consideration. Computer-aided design have introduction in the literature by the research studies which are system specifically designed for the effective and timely development of the design of various projects.

When designing and innovating new products, most designers will use computer-aided innovation technology to complete, integrate various factors into product design, including product design theory, product design mode, innovation technology, computer software technology, and natural language processing technology, and establish a complete computer-aided innovation technology tool and design platform for product design [1]. When using computer-aided innovation technology, designers should first analyze the problems existing during product design, track and mine the problems and system analysis, describe the problems and root causes that should be paid attention to during product design, then further decompose and deal with them, form a problem list, select an ideal treatment scheme, and finally integrate various knowledge resources for product design, risk analysis, and feasibility analysis, and find the ideal alternative and generate the evaluation report [2].

The use of computer-aided technology in production has increased significantly in recent years. With the use of this technology, we may change issues, create methods to solve difficulties, and conduct scientific analyses of problems [3]. The theory of computer-aided innovation technology is being enhanced and implemented in the design of engineering systems, R&D, and product development today. In most businesses, it serves as the primary tool for product design.

The main novelties of this manuscript are given as follows: (1) this paper first summarizes the concept of computer-aided technology, constructs the architecture of computer-aided innovation technology, uses computer-aided technology in the design and assembly of products, and analyzes the assembly relationship of product assembly model. (2) Using the assembly information model diagram to study the conflicts and problems existing in the assembly model, we complete the technological innovation processing of product design through CAI-driven integrated innovation technology, design the assembly model, and use the model to reduce various conflicts in assembly design.

The rest of article is managed as given below.

Literature review of the available techniques is presented in the subsequent section where main stream approaches along with the pros and cons are discussed. The proposed idea of the CAD is described in the section three of the manuscript where initially, it begins with a comprehensive definition (overview) of the respective technology and how it is useful in resolving the problem under consideration in this article. In section four, we have described the CAD and its implementation from the perspective of the problem domain. Results of the simulations under different evaluation metrics have been reported in the section five of the paper. Conclusion and references are presented last in the article.

## 2. Literature Review

In recent years, European and American countries have rapidly developed computer-aided innovation technology (CAI), combined with invention and creation technology and computer software technology, and launched the latest CAI technology. Product design is integrated with an innovation theory and regarded as the core of research and development CAI technology [4]. Vrontis and others emphasized that CAI technology is a key area of computer-aided technology, compiled and analyzed the relevant CAI technology's tools and current state of development, and completed the product optimization design using a combination of market analysis findings and problem-solving techniques, which altered the conventional innovation mode [5]. Supyan et al. utilizing the open innovation approach employed by the corporation in recent years; Cai 2 0 software developed a collectively based intelligent framework, problem-solving process, and collaborative assistance, explored knowledge acquisition, reuse, and capitalization, and tested the method utilizing biomass [6]. Razzaq et al. pointed out the importance of knowledge acquisition and capitalization for innovation and evolution, developed the basic software system based on ontology knowledge acquisition and problem solving, and pointed out that it is necessary to develop innovative software in the field of industrial practice to realize product design [7]. Chen et al. introduced a design optimization algorithm when integrating PLM system and CAI technology, used design optimization algorithm and CAI technology to deal with design conflict, combined with knowledge tools to reuse knowledge, but did not list the basic mechanism combined with KB tools [8]. Deng and Deng pointed out that the PLM system and Cai optimization method can be integrated to improve the product development cycle, and the optimization system is used as the link between the two. During the development of Pro sit project, this method is used to demonstrate the connection procedures and optimization of CAI and PLM system by designing plastic wheels. This integration method reduces the design cost, design problems, and product design efficiency and quality [9]. Te and Wang pointed out that from the perspective of developing new products, he analyzed the development level of CAI technology, proposed to use CAI technology to complete new product development on the basis of information technology and innovative design, discussed and analyzed the potential function, classification and development trend of CAI technology, and pointed out that in the future, CAI technology should be integrated with other technologies in order to provide a more complete product design process for the development of new products [10]. The Yu standard section algorithm, which is used in the software environment, was developed by improving the current standard solution method and solution algorithm. The CAI system, which was developed using this algorithm, uses the algorithm to organize a large number of standard solutions, making the operation more convenient [11]. Song and Zhang CAD software and Cai tools were combined to address the tension between technological advancement and environmental preservation, and the design of ecologically innovative goods was accomplished [12]. Although, these approaches are available in literature and have been used extensively in for solving similar problems like the one we are trying to address in this manuscript, but these approaches are limited to a certain domain and could not be applied to every problem.

## 3. Overview of Computer-Aided Technology

Computer-aided technology (CAT) have been used in the literature for addressing and streamlining the activities where requirements for the computation are relatively higher than existing one. This technology has been adopted for the solving problems related to numerous research domains such as design, integrated modules etc.

### 3.1. Computer Aided-Technology Concept

The basic tool of computer-aided technology is computer, which is the method, theory, and technology used by people in a special field, including computer-aided manufacturing technology (CAM), computer-aided design (CAD), computer-aided instruction (CAI), computer-aided drawing, and computer-aided quality control (CAQ). As a new technology with the fastest development speed in recent years, it is mainly used in enterprise R&D of new products, design process optimization, and manufacturing system. It is a basic tool for innovative product design and process [13]. CAI technology plays an important role in product design and R&D, which can significantly improve the efficiency and quality of product design, assist designers to set out from various scientific fields and use effective technologies and methods to establish scientific and innovative design schemes, greatly improve the efficiency of product design and development, and reduce wasted resources and repeated workload during R&D. In order to significantly increase the effectiveness and capability of enterprise technological innovation, we should first analyze the issues and drawbacks in product process innovation and product design before realizing the innovation of the enterprise in process design, product function, and principle on the basis of problem-solving theory and accumulated knowledge.

For more than 20 years, CAI technology has been created. Many institutions are currently researching the CAI system.  Table 1 lists the primary new software functionalities that are used internationally in this work. The software's theoretical foundation is TRIZ. The product's creative design is finished based on the knowledge effect basis by combining with a range of issue analysis techniques. A detailed explanation of computer-aided innovation in practice is given below.

### 3.2. Computer-Aided Innovation Technology Architecture

The use of CAI technology in the process of product new concept design and scheme design can integrate all kinds of relevant theories, use a large number of website resources to provide technical basis for engineers and technicians, expand the personal concept of designers, facilitate the comprehensive application of all kinds of scientific knowledge, accelerate the innovation process and speed, and get the product design innovation scheme more quickly.  Figure 1 shows the theoretical system of computer-aided innovation. According to Figure 1, during product innovation design, computer-aided innovation technology requires designers to combine with computer technology, input personal creative thinking on the basis of personal experience and resources, so as to provide designers with website resources and knowledge base, and use retrieval technology to assist entrepreneurs in formulating design schemes or ideas.

Enterprises can quickly complete product innovation and development by using the CAI technology, which can significantly reduce the investment cost of enterprises. Using CAI technology can analyze the latest patented technology, reduce the repeated use of other designers' design technology, and better avoid patents; CAI technology can also predict and analyze the development trend of product design technology in the future, so that engineering designers can grasp the advantages of new technology at the first time.

The functional modules in typical CAI software and the characteristics of product innovative design are both thoroughly examined in this paper. Innovative principle, project navigation, other tools for problem-solving, patent search, prediction technology, evaluation scheme, and knowledge management are currently the functional modules of CAI software with perfect functions. These modules may be used by designers to research, analyze, and forecast issues with technological systems and product design, as well as to look at the future direction of product innovation. The rate of mistake in this process can be decreased by creating a logical and scientific product design strategy.

During the process of dealing with problems, designers can use the knowledge of various scientific fields and the experience accumulated by experts on CAI software to find problems in the technical system according to the law of innovation, formulate innovative treatment schemes, and build their own knowledge base and core technology, which can help enterprises avoid existing patent problems and transform patents into independent intellectual property rights.

## 4. Computer-Aided Product Design Technology

This study uses assembly products as the primary research object to advance product design technology and finish the product functional requirements design [14]. It is based on computer-aided research on product design technology. The assembly structure design must complete the product function. The product function structure and product information can be inherited by the assembly structure model, which can then establish a relationship with the product parts. It serves as a foundation for eventual product design, analysis, process planning, and simulation by tightly coupling the product detailed design and conceptual design [15]. The product assembly model may be explained in two different ways: vertical volume level description and horizontal table description. Volume hierarchy description is a vertical logical description used to describe in detail the parent-child relationship between subassembly components, products, parts, and part features of the assembly bidding document. The table description form is used to represent the connection relationship between different structural elements on the same structural layer, which can also be called assembly relationship.

### 4.1. Analysis of Assembly Relationship of the Product Assembly Model

The assembly relationship in the product assembly model is analyzed here, and the assembly model of the assembly relationship is shown in Figure 2. In the Figure 2, it is the assembly drawing of the shaft system components of the reducer subassembly, where UI is the assembly unit, and Figure 3 is the connection diagram of the hierarchical assembly relationship of parts, which belongs to the five-way graph structure of non-connectivity, which is briefly described below.

Suppose the undirected graph is represented by *G*:

(1) $$\begin{array}{c} G=\left(V,E,\Phi \right). \end{array}$$

In the above formula, *V* is a nonempty finite set on vertices, *e* is a finite set of edges, and edges are disordered or ordered pairs on vertices; Φ is the relationship between *E* and *V* elements.

(2) $$\begin{array}{c} V=\left\{v_{1},v_{2},v_{3},v_{4},v_{5},v_{6}\right\},\\ E=\left\{e_{1},e_{2},e_{3},e_{4},e_{5},e_{6},e_{7},e_{8}\right\},\\ \Phi :e_{1}=\langle v_{1},v_{6}\rangle e_{2}=\langle v_{3},v_{6}\rangle e_{3}=\langle v_{2},v_{3}\rangle ,\\ e_{4}=\langle v_{2},v_{6}\rangle e_{5}=\langle v_{2},v_{4}\rangle e_{6}=\langle v_{4},v_{6}\rangle ,e_{7}=\langle v_{5},v_{6}\rangle e_{8}=\langle v_{5},v_{6}\rangle . \end{array}$$

The above formula 〈*v*_1_, *v*_6_〉 is an undirected edge and the endpoints are *v*_1_*V*_1_ and *v*_6_. If there are a large number of assembly units on the assembly, it indicates that the undirected graph has high complexity.

(3) $$\begin{array}{c} G_{i}=\left(V_{i},E_{i},\Phi_{i}\right). \end{array}$$

In the above formula, *V*_*i*_={*v*_1*i*_, *v*_2*i*_, *v*_3*i*_,…}; *E*_*i*_={*e*_1*i*_, *e*_2*i*_, *e*_3*i*_,…}; Φ_*i*_: *e*_1*i*_=〈*v*_1*i*_, *v*_2*i*_〉, *e*_2*i*_=〈*v*_2*i*_, *v*_3*i*_〉, *e*_3*i*_=〈*v*_1*i*_, *v*_3*i*_〉,...; *i* represents the level number.

The following are the basic properties of the hierarchical assembly model of assembly relationship:

1. There is a constraint relationship between different assembly units during the operation of the assembly, and the relationship affects each other.
2. There are many constraints between two different elements, and each edge can represent different constraints.

The vertex objects of an undirected graph composed of different levels in the assembly model are different, and the relationship of corresponding edge composition is also different. The specific contents are listed in Table 2.

Macroscopically, the product function needs to be completed by the assembly structure design, and the micro-perspective analysis should be realized by using the constraints between the features and geometric features between parts. After editing the geometric features and feature constraints, the CAD system can update and realize the editing operation page and ensure the geometric constraint relationship and assembly constraint relationship between products.

### 4.2. CAI-Driven Integrated Innovation Technology

The knowledge-based intelligent system, KBE technology, is widely used in the process of mold design. This technology can improve work quality, improve work efficiency, and store design knowledge [16]. However, KBE technology also has limitations, unable to obtain innovative knowledge, resulting in the lack of innovative characteristics of product design schemes. For this problem, we can make full use of CAI technology to deal with product innovation, add CAI to the innovation idea scheme and output it to KBE, and provide KBE with a new innovation knowledge scheme, so as to obtain, share, and exchange innovation knowledge information.

As a result, by combining semantic processing, CAI, KBE-based knowledge-driven technology, and CAD technology, we can more effectively reflect the benefits of various types of knowledge, fulfil the role of assisting innovative engineering design, conception, and CAD system, and make it easier for quick, innovative product design, and process automation.  Figure 4 illustrates how CAI-driven integrated innovation technology is applied.

The integrated innovation technology should be applied in the conflict resolution principle of TRIZ theory, function cutting, standard solution and geometric effect Cai tools to deal with the design contradiction on the product CAD assembly model, formulate the product design scheme to deal with the contradiction, and then send it to the knowledge-driven automation system (kDa) of UG/NX software. The system uses the absorption mechanism or innovation mechanism to deal with it and constitutes a certain product rule to drive the product structure design, and update the assembly structure model [17, 18].

## 5. Product Design Analysis Results

Examination of the results, preferably of the newly develop technique, is required to be performed prior to its publication. Moreover, especially for the product design, these results should be evaluated extensively or thoroughly to justify claims of the proposed scheme.

### 5.1. Qualitative Analysis Results of Product Design

This paper focuses on computer-aided product design technology, using product design coding rules and segmentation principles to sort out the corpus data in each group of experiments, so as to complete the qualitative analysis of product design [19, 20]. The coding and segmentation contents in this study are shown in Table 3. A-E represents five different designers in each group, and the initial coding of creative points is 0. Selecting two researchers to complete sentence segmentation and coding operations can reduce the subjective interference of a single sentence segmentation to the coder. A large number of creative points can be generated by using oral segmentation and creative coding in oral analysis. Table 3 shows an example of link markers corresponding to oral materials.

Through statistical analysis of the link marking diagrams of test I, II, and III, and listing the link index data in Table 4, there are 58 moves in test I and the number of links is 116. In Experiment II, there were 35 mobile and 70 links. There were 49 movements and 98 links in test III, and the link index Li was 0.6, 0.6, and 0.495, and the Li values of the three groups were generally the same.

There are 14 key movements in test I, 10 key movements in test II, and 11 important movements in test III, according to the test movements in Tables 3 and 4. The brainstorming approach has the highest energy efficiency in product design, while the creative generation structured graphic representation method has the same level of creative energy efficiency as the agitation sketch method, according to the link index and mobile numerical analysis. The statistical entropy results are displayed in Figure 5.

The results of the entropy calculation are treated with the direct method on the link marker maps of the three groups of experiments. The calculated results are shown in Figure 5. The highest direct value of horizontal link is test III and the lowest is test II, indicating that the most active is creative point of III, with the strongest creativity and creativity. The results of experiment I are the highest among the values of front link entropy, while those of experiments II and III are generally the same, indicating that there are more creative points for product design in experiment I. In post-link entropy, experiments I and III are the highest, and their values are basically the same. The lowest is experiment II, indicating that experiments I and III creative points can respond to and improve product design creativity.

### 5.2. Analysis Result of Shaft Assembly Evaluation

In this paper, the effect of product design based on computer aided is evaluated and analyzed from the perspective of shafting assembly system. Before evaluation, each parameter and the evaluation model built should be taken into account [19, 20]. The parameters selected for evaluating the products of shafting assembly system are technical novelty, operation efficiency, assembly accuracy, and input cost. The specific evaluation model is shown in Figure 6.

In the evaluation model established in Figure 6, the main evaluation parameters selected are technological novelty, product operation efficiency, assembly accuracy, and input cost. The product design of shafting assembly system is evaluated. The highest proportion of the ideological parameters is assembly accuracy, accounting for 35%, followed by product operation efficiency, accounting for 25%, and technological novelty for 15%. The proportion of input cost is 25%. After comprehensive evaluation, it is concluded that the product design and assembly accuracy of the shaft assembly system based on computer-aided technology is high, which effectively solves the problem of low traditional assembly situation and greatly improves the assembly efficiency.

## 6. Conclusion

With the rapid development of market economy and the introduction of various products in the market, the competition pressure among enterprises increases. More and more enterprises start from product design to develop new products to improve the competitiveness of enterprises. During product design, computer-aided innovation technology is selected as a tool, which integrates innovation theory, innovation method, and computer technology to continuously improve product design. This paper briefly describes CAI technology-driven technology and establishes an integrated process model, which constructs an assembly information model diagram, analyzes the conflicts and problems in the assembly model, and then uses CAI-driven integrated innovation technology to complete product structure design and implement assembly model design, so as to reduce the conflicts in assembly design. The shafting assembly system product is analyzed by building an evaluation model. According to the selected evaluation parameters, the assembly accuracy of the product reaches 35%, the input cost is 25%, the technical novelty accounts for 15%, the product operation efficiency is 25%, and the proportion of each parameter is balanced, which can give full play to the product advantages.

## Figures and Tables

**Figure 1:** CAI framework system.

**Figure 2:** Shafting assembly structure.

**Figure 3:** Assembly diagram.

**Figure 4:** Application process of CAI-driven integrated innovation technology.

**Figure 5:** Entropy calculation results.

**Figure 6:** Evaluation model.

**Table 1:** CAI software statistics.

Number	Software name	Major function	Development company	Composition knowledge base
1	Pro/Innovator	Integrate natural language processing technology, invention and creation, computer software technology, etc., including system analysis, project navigation, problem decomposition, creation principle and scheme evaluation	IWINT Inc	Effect base, case base, patent query and user knowledge base

2	Goldfire Innovator	Provide systematic and comprehensive solutions for engineers to deal with innovation problems, involving modules such as researcher, innovator, analysis of innovation trend, innovation resource base and knowledge management system	Invention Machine Corporation	Patent database, scientific effect database and examples, patent website, personal knowledge database and enterprise knowledge database

3	Innovator Work Bench(IWB)	Provide engineers with a structured way to solve innovation problems. The modules involved include problem expression, problem analysis, system operation, e-learning module, evaluation, innovation case base, and navigation	Ideation International Inc	Patent website, effect database, examples

4	CREAX Innovator	Assist engineers to complete innovation and deal with conflicts according to the process. The modules involved include description problems, definition problems, system model, idealization, selection tools, contradiction matrix, innovation principle, knowledge tools, understanding map, conception management and evaluation tools	CREAX NV	Online patent library, USA and Canada, professional website search, function library

**Table 2:** Table relationship between vertices, edges, and objects in hierarchy.

	Model hierarchy	Vertex	Edge
*i* = 1	Assembly layer	Root node	--
*i* = 2	Subassembly layer	Subassemblies and parts	Assembly relationship between subassembly and parts
*i* = 3	Part layer	Spare parts	Assembly relationship between parts
*i* = 4	Assembly feature layer	Spare parts	Constraint relation and adjacency relation between geometric features
*i* = 5	Geometric topology layer	Geometric features	Adjacency relationship between different geometric elements

**Table 3:** Segmentation and coding examples.

Creative coding		Oral materials	Idea
A	0	What is the sliding bearing structure used in the front bearing system of the main shaft?	Front bearing structure of main shaft
	1		Sliding bearing
B	2	Can the temperature be reduced or meet the requirements of high-speed rotation?	Low spindle component temperature
	3	I do not think so	High speed rotation of spindle
C			--
D	4	Usually, the spindle rotating at high-speed uses rolling bearings, which will reduce the spindle temperature	Rolling bearing
E	5	I agree that zqsn is usually selected as the sliding bearing material, which is difficult to maintain in the later stage	Sliding bearing material
	6	Yes, it is difficult to adjust the clearance of this type of bearing. If the clearance is set too high, it cannot meet the accuracy requirements	Bearing maintenance
B	7		Adjust bearing clearance
	8	If the gap is small, it will lead to excessive heating	Accuracy requirements
A			--
B	9	It will increase the degree of bearing wear and the spindle temperature will also rise	Bearing wear

**Table 4:** Link index statistics.

	Ideas/moves quantity	Number of links	Link index *L*1
Test 1	58	117	0.6
Test 2	35	71	0.6
Test 3	49	98	0.495

## Data Availability

The datasets used during the present study are available from the corresponding author upon reasonable request.
